This article has been retracted.

# Application of RoboCup 3D and Intelligent Technology in Football Simulation League

**DOI:** 10.1155/2022/9676952

**Published:** 2022-07-09

**Authors:** Shenghui Wei, Huibing Qin

**Affiliations:** ^1^School of Physical Education and Health Sciences, Chongqing Normal University, Chongqing 401331, China; ^2^Institute of Physical Education, Hubei University of Science and Technology, Xianning, Hubei 437100, China

## Abstract

Intelligent technology has been recently more developed which is due to the advancement in the technology sector. Moreover, every industry is now moving toward adoption of the intelligent technology to provide better services along with informed decisions which are possible only if devices have built-in intelligence. Likewise, in football simulation league, assigning suitable roles to each robot according to the real-time characteristics of complex and changeable field conditions is the key to win the game. In order to solve the problems of low research efficiency and poor simulation effect, this paper aims to deeply explore the application of RoboCup 3D and intelligent technology in football simulation league. Firstly, the movement speed, shooting speed, and direction of the players are measured. Secondly, a highly intelligent goal keeping and defense method and triangle attack strategy are proposed. The defense strategy is mainly that when the other team is in the state of attack, we send players to intercept the other player with the ball, and the triangle attack strategy is to use the three players in the appropriate position to cooperate with each other. The triangular attack team is composed of core attacking players and two auxiliary attacking players. This method is applied to football simulation league. RoboCup 3D simulation experiments show that the proposed method has good simulation effects in terms of ball loss rate and winning streak, which shows that the proposed method can effectively improve the research efficiency and simulation effect and has certain practicability.

## 1. Introduction

RoboCup 3D simulation robot soccer game mainly provides a research platform for an autonomous agent system to simulate the actual football field. At an interval of 20 ms, the robot obtains some information such as the status of the court and the shouting of teammates through server communication. In the process of the game, in order to significantly optimize the overall team ability, having an efficient robot system is the key to the team's victory. According to experience, if we use the allocation of role positions to ensure the formation and formulate a democratic voting mechanism to unify the decision-making of the whole team on the playing field, we can not only make the team more orderly as a whole but also effectively play the offensive and defensive ability of different roles. The robot football World Cup's principal goal and significance are very obvious. It can encourage the advancement and development of robot and artificial intelligence, as well as certain associated scientific studies, through the world's most popular sport, football. Technology integration and breakthroughs, such as physical sensors, artificial intelligence, and energy storage, are required to achieve behaviors such as robot dribbling, passing, and kicking. More inventions and new achievements are bound to emerge as a result of the long-term goal of a robot playing football, and these high and new technologies are widely used in many industrial production fields and life fields, such as construction engineering, transportation, and wireless communication, to meet the wide needs of the public. Therefore, this paper makes an in-depth study on the application of RoboCup 3D and intelligent technology in the football simulation league.

The innovations of this paper are as follows: (1) We calculate the movement speed, shooting speed, and direction of players and then put forward a high intelligent goal keeping and defense method and triangle attack strategy. (2) RoboCup 3D simulation experiments show that the proposed method has good simulation effect, can effectively improve the efficiency of research, reduce the economic cost of research, and has certain practicability.

The remaining paper is given as follows: in the Related Work section, we have tried to explain what actually is available in the literature related to the problem domain and what are the issues associated with these techniques. What is the main problem which is needed to be resolved on priority basis?

## 2. Related Work

In recent years, researchers at home and abroad have carried out various research studies on robot football under different backgrounds and achieved corresponding results. In order to effectively improve the efficiency of intelligent cooperation and enable the robot football team to achieve better competition results, Hang and Fang proposed an agent system cooperation mechanism based on the hierarchical model. The layered model specifically includes the main communication layer of agent communication, the role allocation technology layer of agents, formation positioning, and other decision-making control layers. The simulation results show that team cooperation is the focus of scoring in robot football game. The cooperation mechanism based on the hierarchical model plays a significant role in improving the overall confrontation ability of robot teams, but this method is not practical [1]. The in-depth analysis of football game analysis method based on location data, according to Wang and You, can find that the team center can clarify the geometric center of the team, the spatial control method can calculate the player coverage area, the network analysis method can measure the passing behavior of the team, and the machine learning algorithm can identify the tactical characteristics of the team. While location data are merely big data in a single spatial mode, big data technology is promoting a new revolution in the field of football study. Subsequent research should use the integration of training needs, cycle load, and players' physical fitness to compress location, psychology, and coach data into relatively small variables and use the simulation environment to optimize the prediction of sports performance results to a certain extent, but this method is more complex and it leads to the poor effect of football simulation competition [2]. Liao et al. proposed that in the process of soccer robot movement, soccer robots are mostly in the environment of real-time confrontation. Therefore, robots must have relatively high ability to cope with the movement process. For every important moment, such as the process of robot grabbing the ball or the process of robot controlling the ball, we need to make a scientific response. Most strategy studies only focus on the path planning of the robot in the process of ball control but do not comprehensively consider the process of robot competition, resulting in the lack of key links in the process of football robot movement, the loss of integrity, and the neglect of real-time confrontation. Therefore, the competition model of WTA is used to solve the competition problem of robot, and then, the improved path planning method is adopted to avoid obstacles. The disadvantages of traditional path planning algorithms are effectively solved, and the efficiency is improved. Simulation experiments show that the method is correct, but the scientificity and practicability of the method have not been verified [3]. Yu analyzes that the gait instability of the leg mechanism of the soccer robot will occur when it is disturbed by the zero-torque point. As a result, a dynamic model of a robot limb based on vibration suppression and an optimum control rule is provided. The dynamic model successfully identifies the mechanical characteristics of the robot leg, and the walking vibration suppression and the control law model, as well as the uncoordinated state space model, are developed. To accomplish integrated control of the leg mechanism and gait planning of the football robot, the tracking error technique and feedback adjustment method are employed to construct the optimal control law. The simulation results reveal that this method's design effect and gait planning stability are generally excellent, and its tracking adaptive adjustment ability is great although it has some tracking error [4].

## 3. Measurement of Players' Movement Direction, Shooting Speed, and Shooting Direction

The motion of a soccer robot may be divided into three categories: motion direction, speed, and kicking. Three motion parameters are calculated to indicate robot decision-making [5, 6]. For simplicity, these are explained in different subsections which are given as follows.

### 3.1. Measurement of Robot Motion Direction and Speed

The robot can use the positioning system and communication system to obtain its own position with the football. The movement direction of the robot to the football is calculated and expressed as follows:

(1) $$\begin{array}{c} \text{arctan}\frac{d_{y}}{d_{x}}. \end{array}$$

Here, *d*_*x*_ represents the abscissa difference between two points on the court and *d*_*y*_ represents the difference of ordinates between two points on the court.

The speed of the robot mainly depends on its current position and its own characteristics. When the robot is picked up at the nearest location to the offensive, the speed of robot follows as the fastest (*V*_*f*_); otherwise, it moves to the football according to the speed of energy-saving roaming (*V*_*n*_). In this study, the relationship between *V*_*f*_0 and *V*_*n*_ is represented as follows:

(2) $$\begin{array}{c} V_{f}=2V_{n}. \end{array}$$

### 3.2. Direction of Soccer Robot Kicking (*α*) and Speed Measurement

The robot has the idea of kicking the ball to the opponent's goal, so it hopes to kick the ball into the opponent's goal every time it plays football. It is also because the robot has this idea that the robot has running power, but in fact, there are some differences between the idea and the actual effect. Therefore, the random deviation value (*η*) is inserted in this paper. Because the random deviation value (*η*) makes the difference between the league process and the result, which cannot be predicted, this increases the suspense of the game [7, 8]. Therefore, the data model for the measurement of kicking direction (*α*) is expressed as follows:

(3) $$\begin{array}{c} \alpha =\arctan\frac{g_{x}-x}{g_{y}-y}. \end{array}$$

Here, *g*_*x*_ represents the abscissa position of the goal, *g*_*y*_ represents the ordinate position of the goal, *x* represents the abscissa position of the ball robot, and *y* represents the ordinate position of the ball robot.

In order to make the football operation closer to the real situation, a speed mathematical model is set for the football. In the model, the football speed is related to the shooting ability of the robot and the running speed at that time. The specific model is expressed as follows:

(4) $$\begin{array}{c} v=\left(\frac{S_{p}}{2}+n\right)\times S_{v}. \end{array}$$

Here, *S*_*p*_ represents the fastest speed of the robot shooting, *S*_*v*_ represents the fastest speed of the robot approaching the football, and *n* represents a random quantity [9, 10].

### 3.3. Measurement of Distance between the Robot and Football

The distance between the robot and the soccer ball is a factor in the robot's real-time calculations. The computation frequency is rather high, and the real-time performance is quite good. As a result, the number of calculations is decreased. This study investigates the mathematical model of formula (5), which performs just the addition and subtraction methods without multiplication or square computation in order to save calculation time:

(5) $$\begin{array}{c} {\text{d}}_{s}=\left|R_{x}-F_{x}\right|+\left|R_{y}-F_{y}\right|. \end{array}$$

Here, *R*_*x*_ represents the position of the abscissa of the soccer robot, *R*_*y*_ represents the position of the ordinate of the soccer robot, *F*_*x*_ represents the position of the abscissa of the soccer robot, and *F*_*y*_ represents the position of the ordinate of the soccer robot.

## 4. RoboCup 3D and Intelligent Technology in Football Simulation League

Intelligent technology has been used extensively in various application areas throughout the world with specific emphasis on how this technology will enhance the operational capabilities of the existing approaches or basically improve both precision and accuracy ratios of the decision models.

### 4.1. Robot Goalkeeper Defense Strategy

Key is defined as the coordinate point that the current goalkeeper needs to reach. The Key value is the trade-off value between *K*_*b*_ and *K*_*q*_. The distance between the opponent's striker and the ball can calculate the probability that the ball is in the shooting state or nonshooting state. Therefore, the distance *d*_*qb*_ between the opponent's striker *R*_*q*_ and ball *B* is expressed as a trade-off factor. If the distance between the opponent's striker and the football is far away, the probability that the football is in the shooting state is relatively high and the Key is closer to the point *K*_*b*_. When the opponent's forward is close to the football, the probability that the football is in the state of nonshooting is relatively high and Key is closer to the point *K*_*q*_. Therefore, it can be concluded that the motion model of goalkeeper defense is as follows:

(6) $$\begin{array}{c} \text{Key}=K_{b}\times \frac{d_{pb}}{R}+K_{q}\frac{\left(R-d_{qb}\right)}{R}. \end{array}$$

Formula (6) solely evaluates the impact of the distance between the opponent's striker and the football on the shooting state; however, it is insufficient. In actuality, the relative pace of the opponent's striker during dribbling and football will alter the shooting state of the ball [11, 12]. Although the distance between the opposition striker and the football is less, their speeds are diametrically opposed. To bring the point near to the key, we use formula (6). There is no collision in reality. The defense collapses if the football is ran to. As a result, the factor is introduced as the trade-off factor using formula (6). The higher the value of *V*_1_, the higher the chance of a nonshooting state. The smaller the value of *V*_1_, the smaller the possibility of nonshooting state. *V*_1_ is expressed by solving

(7) $$\begin{array}{c} V_{1}=V_{q}\times \;\cos\;a-V_{b}. \end{array}$$

In formula (7), *V*_*q*_ represents the speed of the opponent's forward, *V*_*b*_ represents the football speed, and *a* represents the included angle of the walking path. After improvement, the goalkeeper's motion model is expressed as follows:

(8) $$\begin{array}{c} \text{Key}=K_{b}\times \frac{t_{qb}}{t_{k}}+K_{q}\times \frac{t_{k}-t_{qb}}{t_{k}},\\ t_{qb}=\frac{d_{qb}}{V_{1}}. \end{array}$$

Here, *t*_*k*_ represents the coefficient of sensitive time. Due to the difference of the threat of football to the goal in different areas on the pitch, the value of the coefficient *t*_*k*_ of sensitive time is different and the optimal value model can be found in the process of practice. *t*_*k*_ determines the radius *R* of the sensitive area, which is expressed as follows [13, 14]:

(9) $$\begin{array}{c} R=f\left(t_{k}\right). \end{array}$$

Formula (8) is used for defense. Formula (8) comprehensively considers the influence of the distance between the opponent's striker and the football, the running direction of the football, and the relative speed of the football on the shooting state and connects the goalkeeper's running position Key with the two shooting Key points, so as to make the goalkeeper gradually approach the Key points with high probability, coordinate and smooth the movement turn, and finally complete the main purpose of successful defense [15, 16].

### 4.2. Triangle Attack Strategy

Figure 1 shows the implementation process of the triangle attack strategy. The triangle attack strategy mainly takes the football coordinate position as the decision reference and judges the situation on the court according to the football position. If we judge that we are in the state of ball control, we can carry out the attack strategy; otherwise, we can adopt the defensive strategy. In the process of implementing our attack strategy, we must obtain the coordinates and hitting angle of the player's position according to the position relationship between the football and goal, then select the triangular attack of core attacking player and auxiliary attacking player, and then implement the decision [17, 18].

#### 4.2.1. Schematic Diagram of Offensive Shooting

The shooting diagram of triangle attack strategy is shown in Figure 2. The most critical ability of attack is shooting and scoring, and the success rate of shooting is an important factor affecting the goal.

In Figure 2, the black circle is the defensive player of the other side, the red circle is the offensive player of our side, and the black rectangle represents the goal of the other side, which represents the shot − success(*d*, *e*, *f*, *g*) success rate as follows:

(10) $$\begin{array}{c} \text{shot}-\text{success}=\frac{1}{g+1}\times \left\{\frac{1}{{\left(1+d\right)}^{2}}\frac{e}{\pi }+\frac{ef}{f_{\max}\left(1+d\right)\pi }\times 1-\frac{1}{{\left(1+d\right)}^{2}}\frac{e}{\pi }\right\}. \end{array}$$

Here, d represents the nearest shooting distance, *e* represents the shooting angle of the attacking player, *f* represents the index of the attacking player's ability, and *g* represents the interference factor of the defensive player.

(11) $$\begin{array}{c} e=\frac{\arccos\left[\left(p_{1}-p\right)\left(p_{2}-p\right)+\left(q_{1}-q\right)\left(q_{2}-q\right)\right]}{\sqrt{\left(p_{1}-p\right){\left(q_{1}-q\right)}^{2}}\times \sqrt{{\left(p_{2}-p\right)}^{2}{\left(q_{2}-q\right)}^{2}}}. \end{array}$$

Here, (*p*, *q*) represents the position coordinates of the attacking player, and (*p*_1_, *q*_1_) and (*p*_2_, *q*_2_) represent the coordinates of the positions of the two goals.

#### 4.2.2. Player Role Assignment

According to the position, hitting, and angle of players and football, we select the core offensive players and auxiliary offensive players and define the important defensive players of the other party and the goal and ball of the other party as *a*, *b*,  and *c*. The selection of players for core attack is shown in Figure 3.

In Figure 3, the relationship between our three members and the football position and hitting angle is shown as follows:

(12) $$\begin{array}{c} \left(\begin{array}{c} k_{1}=\mu \sigma_{1}DH_{1}c+\sigma_{2}\alpha \\ k_{2}=\mu \sigma_{1}DH_{2}c+\sigma_{2}\beta \\ k_{3}=\mu \sigma_{1}DH_{3}c+\sigma_{2}\gamma \end{array}\right). \end{array}$$

Here, *μ* represents a constant that places distance and angle on an order of magnitude. *σ*_1_ and *σ*_2_ represent the weighted correlation coefficient, which mainly reflects the key to attack of the distance and angle between our players and football. *σ*_1_+*σ*_2_=1, *DH*_1_*c*, *DH*_2_*c*, and *DH*_3_*c* represent the distance between our attackers and football; *α* and *β* and *γ* represent the direction of our attackers'action and the angle between players' connections.

In Figure 4, the relationship between our two players and the main defensive players of the other party and the central position of the other party's goal is shown as follows:

(13) $$\begin{array}{c} \left(\begin{array}{c} k_{4}=\sigma_{1}DH_{2}a+\sigma_{2}DH_{2}b\\ k_{5}=\sigma_{1}DH_{3}a+\sigma_{2}DH_{3}b \end{array}\right). \end{array}$$

Here, *σ*_1_ and *σ*_2_ reflect the importance of distance between our players and their opponent's defenders and their goal centers for the selection of key assistants [19, 20]. *DH*_2_*b* and *DH*_3_*b* represent the distance between our players and the center of the opposing goal [21].

#### 4.2.3. Player Action Selection

The core offensive player performs dribbling, passing, and shooting actions, and the influencing factors on the action selection of the core offensive player are shown in Figure 5.

The variables that affect the player's action choice of core attack are defined as input variables, expressed as follows:

(14) $$\begin{array}{c} \left(\begin{array}{c} m_{1}=I_{1}=\frac{\text{d}x}{\text{d}y}\\ m_{2}=I_{2}=\frac{\text{d}x_{1}}{\text{d}y_{1}}\\ m_{3}=\mu \sigma_{1}Dbc+\sigma_{2}\theta_{bc}\\ m_{4}=\mu \sigma_{1}DH_{1}b+\sigma_{2}\theta_{bH_{1}}\\ m_{5}=\mu \sigma_{1}DH_{2}b+\sigma_{2}\theta_{bH_{2}}\\ m_{6}=\mu \sigma_{1}DH_{1}a+\sigma_{2}\theta_{aH_{1}}\\ m_{7}=\mu \sigma_{1}DH_{2}a+\sigma_{2}\theta_{aH_{2}} \end{array}\right). \end{array}$$

Here, *m*_1_ represents the probability that a core attacker's goal will be intercepted by his opponent's goalkeeper. *m*_2_ represents the probability that a core attacker's goal will be intercepted by his opponent's goalkeeper when he passes the ball. d*x* represents the central connection of the opposing goalkeeper to the opposing goal; d*x*_1_ represents the distance from the opposing defender to our assistant attacker; d*y* and d*y*_1_ represent the distance from the football to the foot. *m*_3_ represents the center position and angle relationship between the football and the opposing goal; *m*_4_ represents the central position and angle relationship between the core attacker and the opposing goal; *m*_5_ represents the central position and angle relationship between the assistant attacker and the opposing goal. *Dbc* denotes the center distance between a football goal and the opposing goal; *DH*_1_*b* represents the center distance between the core attacker and the opposing goal; *DH*_2_*b* represents the center distance between the assistant attacker and the opposing goal; *θ*_*bc*_ stands for the angle between the center of the football goal and the other goal; *θ*_*bH*_1__ represents the angle between the core attacker and the center of the opposing goal. *θ*_*bH*_2__ represents the angle between the assistant attacker and the center of the opposing goal; *m*_6_ represents the position and angle relationship between the core attacker and the opposing defender; *m*_7_ represents the position and angle relationship between the assistant attacker and the opposing defender; *DH*_1_*a* represents the distance between the core attacker and the opposing defender; *DH*_2_*a* represents the distance between the assistant attacker and the opposing defender; *θ*_*aH*_1__ represents the angle between the core attacker and the opposing defender; *θ*_*aH*_2__ represents the angle between the assistant attacker and the opposing defender. We complete the football simulation by the above process.

## 5. Analysis of Experimental Results

In order to verify the performance of the proposed method in football simulation league, experiments are carried out on the simulation platform.  Table 1 shows the experimental data.

On the RoboCup 3D simulation platform, two models, the model proposed in this paper and the traditional model, are selected for 30 simulation games. Each time, the position of the football is changed, and the average planning time, the number of dead cycles, and the number of successes are recorded. The results are shown in Table 2. It can be seen from Table 2 that the model proposed in this paper takes less time to complete the same task and the success rate is relatively high, which can effectively reduce the number of times the model enters the dead cycle, so as to improve the effect of football game simulation.

Two different role assignment methods are used for 30 matches.  Figure 6 shows the comparison of the goal difference results between the method proposed in this paper and the method based on behavioral role assignment.  Table 3 shows the statistical results of the experimental data of the proposed method and the behavior role assignment method.

It can be seen from the data in Figure 6 that the method proposed in this paper can effectively improve the efficiency of goals. In this study, the average difference target is 1.63 and the behavior role-based allocation technique is 1.28. As a consequence, it can be concluded that the strategy suggested in this research is practical, meets the requirements of simulated league matches, and produces good results. Because of the extensive examination of the job allocation criteria, the approach provided in this research makes role allocation more rational, as shown in Table 3. At the same time, the role distribution plan may be changed at any moment to ensure that the robot has a lengthy ball control time and that the team can play better in both defense and offence in simulated leagues and reduce the economic cost of research.  Figure 7 shows the comparison between the proposed method and the traditional method in 30 football simulation matches.

Through the analysis of Figure 7, it can be seen that the ball loss rate of the simulation game of the traditional method increases with the increase in the number of games, while the ball loss rate of the method proposed in this paper is relatively low from the beginning of the simulation game. With the increase in the number of simulation games, although it fluctuates slightly, the overall ball loss rate is low, which shows that the effect of the football simulation league using the method proposed in this paper is better.

## 6. Conclusion

Through the soccer robot simulation soccer game system, the computer screen is used as the venue of the football league and the soccer robot is simulated as an agent to effectively solve the problems of high competition cost and great difficulty of the soccer robot. In the process of practical application, the physical soccer robot game can be effectively verified in the RoboCup 3D game system and applied to the physical robot game after reaching the corresponding expected goal. The method proposed in this paper can effectively improve the efficiency of research and reduce the economic cost of research, which shows that this method is effective and practical.

## Figures and Tables

**Figure 1:** Flow chart of the triangle offensive strategy.

**Figure 2:** Shooting diagram.

**Figure 3:** Core offensive player selection chart.

**Figure 4:** Main auxiliary offensive player selection chart.

**Figure 5:** Factors influencing the action selection of core offensive players.

**Figure 6:** Comparison of statistical results of goal difference in different kicking methods.

**Figure 7:** Comparison of the ball loss rate in football matches with different methods.

**Table 1:** Experimental data.

The experimental configuration	Data
The simulation platform	SimSpark
The game environment	RoboCup 3D
Computer server	BIM computer

**Table 2:** Model strategy comparison of different methods.

Indicators	The traditional model	The model proposed in this paper
Planning time/s	35.3	27.1
Number of successes	41	47
Number of dead cycles	3	1

**Table 3:** Statistical table of experimental results of simulation competition.

Comparison of the item	Behavior-based role assignment approach	The method proposed in this paper
Wins	41%	59%
Goals	87	137
Scoring rate	10.3%	35.7%
Possession	31.3%	68.7%
Average time spent on role assignment	158 ms	141 ms

## Data Availability

The datasets used and/or analyzed during the current study are available from the corresponding author on reasonable request.
